# Effect of Chaihu Shugan Pills on the Pharmacokinetics of Duloxetine and its Metabolite 4-Hydroxyduloxetine in Beagle Dogs: A Herb-Drug Interaction Study

**DOI:** 10.1155/2022/2350560

**Published:** 2022-08-17

**Authors:** Yun-tian Bi, Yao-ren Kang, Ghulam Woshur, Hao-zhe Ding, Shan-shan Wang, Xiang-jun Qiu

**Affiliations:** School of Basic Medical Sciences, Henan University of Science and Technology, Luoyang 471023, China

## Abstract

The effect of Chaihu Shugan pills (CHSG) on the pharmacokinetics of duloxetine and its metabolite 4-hydroxyduloxetine in beagle dogs was investigated by establishing an ultra-performance liquid chromatography-tandem mass spectrometry (UPLC-MS/MS) method to simultaneously measure the concentrations of duloxetine and 4-hydroxyduloxetine in beagle dog plasma. Duloxetine and 4-hydroxyduloxetine were separated on the UPLC-C18 column after acetonitrile precipitation and detected by mass spectrometry with multireaction detection mode (MRM). Six adult healthy beagle dogs (weighing 7–9 kg, male and female) were randomly selected and examined for a single-dose administration of duloxetine hydrochloride (2 mg/kg, control group) and oral administration of CHSG (0.3 g/kg) twice daily for 15 consecutive days followed by a single-dose administration of duloxetine hydrochloride (2 mg/kg, experimental group) using the self-control method. All plasma samples were treated in the same way, and then the concentrations of duloxetine and 4-hydroxyduloxetine were determined using the established UPLC-MS/MS method. The obtained data were subjected to DAS 2.0 software to calculate the pharmacokinetic parameters, and SPSS 20.0 software was used to compare the differences between the two groups. Duloxetine and 4-hydroxyduloxetine had a good linear relationship in the ranges of 1–1000 ng/ml and 0.1–100 ng/ml, and the lower limits of quantification (LLOQ) were 1 ng/mL and 0.1 ng/ml, respectively. The precision, accuracy, extraction recovery, matrix effect, and stability meet the requirements of the guiding principles. After combination with CHSG, *C*_max_ and AUC_0⟶t_ of duloxetine decreased by 49.33% and 13.08%, respectively, and *t*_1/2_ was shortened to 10.17 h; *C*_max_ and AUC_0⟶t_ of 4-hydroxyduloxetine decreased by 71.47% and 48.78%, respectively, and *t*_1/2_ was shortened to 7.97 h. The UPLC-MS/MS method was fully developed to simultaneously measure the plasma concentration of duloxetine and its metabolite 4-hydroxyduloxetine in beagle dogs. CHSG could slow down the absorption of duloxetine, induce the metabolism of duloxetine and 4-hydroxyduloxetine in beagle dogs, and reduce plasma exposure.

## 1. Introduction

Depression, also known as melancholia, is a clinical manifestation of anxiety, cognitive impairment, and hallucinations. Chaihu Shugan Pills (CHSG) originated from Jing Yue Quan Shu in Ming Dynasty and had been widely used in clinical practice. The information on components in CHSG is shown in Figure 1 and Table 1. The combination of these drugs had anti-inhibitory depressive effects [1], modulation of a hypolipidemic and neuroendocrine-immune network [2], anti-inflammatory and antioxidative stress [3], and hypoglycemic and antifibrotic pharmacological effects [4].

As a safe adjuvant alternative therapy, CHSG in combination with other chemotherapy regimens could improve the therapeutic effect, reduce the bone marrow suppression caused by chemotherapy drugs, and improve the healing of breast cancer patients [5]. Because of its effect of draining the liver and strengthening the spleen, activating blood circulation, and relieving depression, it could alleviate the loss of liver health caused by emotional factors. CHSG was effective and safe in treating depressed patients [6]. Through releasing the inhibition of the Gria3 and MAPK14 signaling pathways, CHSG exerted an antidepressant-like effect by downregulating miR-124 expression [7].

Duloxetine hydrochloride (Figure 2(a)) is a 5-hydroxytryptamine (5-HT) and norepinephrine (NE) reuptake inhibitor which has a relatively weak inhibitory effect on dopamine reuptake. Originally approved by the U.S. Food and Drug Administration (FDA) in 2004 for the treatment of major depressive disorder (MDD), duloxetine hydrochloride is currently approved in many countries for the treatment of generalized anxiety disorder (GAD), diabetic peripheral neuropathic pain, fibromyalgia (FM), and chronic musculoskeletal pain and, in Europe, for the treatment of stress urinary incontinence [5]. After entering the body, duloxetine was metabolized by the isoenzymes 2D6 and 1A2 of CYP450 [6], and the main metabolite was 4-hydroxyduloxetine (Figure 2(b)). Duloxetine hydrochloride had good efficacy in depression but was often accompanied by numerous adverse effects: iris relaxation syndrome, hypertension, hyponatremia, Parkinson's syndrome, 5-hydroxytryptamine syndrome, increased risk of traumatic brain injury in the elderly, and so forth [7]. Therefore, it was of abysmal clinical significance to find a safe, effective, and fewer-side-effects way of administration when using duloxetine for clinical treatment.

With the wide application of traditional Chinese medicine, the mode of combining Chinese and Western medicines has provided new ideas for clinical treatment. A large number of studies had demonstrated that the combination of Chinese and Western medicines could improve the efficacy of Western medicines and reduce toxic side effects at the same time [8–10].

Currently, CHSG combined with duloxetine hydrochloride is also used in clinical practice. The efficacy of a single-dose group (duloxetine hydrochloride) versus a combination group (duloxetine hydrochloride combined with CHSG plus and minus formula) on depression was evaluated, and the results showed that the combination group had better efficacy and a lower incidence of concomitant adverse effects, which was worth promoting in the clinic. CHSG in combination with duloxetine was used for the treatment of Parkinson's depression, which could not only improve the manifestations of depression but also improve the cognitive ability of patients, and its clinical efficacy was better than that of single-dose duloxetine [11]. Due to the regulation of the BDNF/ERK/CREB signaling pathway in the hippocampus and frontal cortex, CHSG and coadministration of CHSG and fluoxetine could relieve and improve depression-like behavior and cognitive function. The coadministration of CHSG and fluoxetine could enhance the antidepressant effect of CHSG and fluoxetine alone, and there might be a drug interaction between CHSG and fluoxetine [12].

The combination had achieved good results in clinical practice, but the safety of the combination was unclear and had not been reported at home or abroad. Therefore, to provide some basis for their safe use in clinical practice, we selected 6 beagle dogs and compared the changes in the pharmacokinetics of duloxetine given in a single dose with those of duloxetine given after 15 days of continuous administration of CHSG and investigated the effects of CHSG on duloxetine and 4-hydroxyduloxetine using a self-control method. We hope that our study could provide some scientific basis for the safety of the combination of CHSG and duloxetine hydrochloride in clinical practice and also provide some guidance for the rational combination of Chinese and Western drugs.

## 2. Materials and Methods

### 2.1. Chemicals Materials

CHSG were purchased from Pujitang Pharmacy (batch numbers: State Drug Quantifier Z13020690, Z13020687, and Z13020702). Duloxetine hydrochloride enteric-coated tablets were purchased from Jiangsu Enhua Pharmaceutical Company Limited (lot no.: State Pharmaceutical Code H20130056).

Duloxetine standards were purchased from Shanghai Jizhi Biochemical Technology Co., Ltd. (purity: 98%, CAS: 136434-34-9, lot number: D66280). 4-Hydroxyhydroxylate standards were purchased from Yongcheng Pharmaceutical Technology (Huangshi) Co., Ltd. (purity: 94.8%, CAS: 662149-13-5, lot number: 392524D). Fluoxetine (internal standard, IS) standards were purchased from Shanghai Maclean Biochemical Technology Co., Ltd. (purity: 99%, CAS: 59333-67-4, lot number: F830634).

Chromatographically pure acetonitrile and methanol were purchased from Merck (Darmstadt, Germany).

### 2.2. Instruments

Waters ACQUITY UPLC I-Class was used as the chromatographic separation instrument, including quaternary solvent manager, sample manager-flow through a needle, and high-temperature column heater with active preheating (Waters, USA).

Waters XEVO TQD triple quadrupoles mass spectrometer was used as the mass spectrometer and the electrospray ionization (ESI) source was used (Waters, USA). Other instruments included ultra-pure water equipment, vortex mixer, and electronic analytical balance.

### 2.3. Animal Experiments

Six healthy beagles (3 males and 3 females, weighing 7–9 kg) were fed in a laboratory with a temperature of 25°C and 12 hours of light, humidity-controlled at 38%–65%, fed twice a day, and fasted for 12 h before the experiment, with no restriction on water intake. The animal license number is SCXK (HUBEI) 2016–0020. All animals were provided by the animal laboratory of Henan University of Science and Technology (Luoyang, China) and authorized by the animal ethics committee of the animal laboratory of Henan University of Science and Technology.

Six beagle dogs were weighed before the experiment, and duloxetine hydrochloride enteric tablets (control group) were administered orally at 2 mg/kg on the day of the experiment, followed by 10–20 mL of saline to ensure complete entry of the drug into the body. After administration, 1 mL of venous blood was drawn from the small saphenous vein of the forelimb at 0.5, 1, 1.5, 2, 3, 4, 6, 8, 12, 24, 36, and 48 h and placed in heparinized EP tubes. The samples were then centrifuged at 10,000 rpm for 10 min, and the plasma was removed and stored at −20°C, pending measurement.

After a one-week drug washout period, CHSG 0.33 g/kg was given orally twice daily for 15 days. On the morning of the 16th day, 2 mg/kg of duloxetine hydrochloride enteric tablets (experimental group) was given transorally half an hour after the administration of CHSG. Blood samples were also collected at 0.5, 1, 1.5, 2, 3, 4, 6, 8, 12, 24, 36, and 48 h and processed according to the same conditions as above.

### 2.4. Analytical Conditions

The Column YZZsed in the experiment was an Acquity BEH C18 column (2.1 mm × 50 mm, 1.7 *μ*m), maintained at 45°C, with a total analysis time of 2 min. The mobile phase A was 0.1% formic acid and B was acetonitrile and the gradient elution procedure is shown in Table 2. The mass spectra were performed in multiple reaction monitoring mode (MRM) under positive ion conditions with an ESI source. The parent ions and daughter ions used for quantitative detection were m/z 298.2⟶157.2 for duloxetine, m/z 314.3⟶124.2 for 4-hydroxyduloxetine, and m/z 310.2⟶44 for Is, respectively.

### 2.5. Solutions Preparation

10 mg of duloxetine standard was precisely weighed and dissolved fully in methanol and the volume was fixed to 10 mL to obtain 1 mg/mL of duloxetine stock solution.

10 mg of the 4-hydroxyduloxetine standard was precisely weighed and dissolved in methanol with volume to 10 mL to obtain 1 mg/mL of 4-hydroxyduloxetine stock solution. Fluoxetine (IS) standard 10 mg was weighed and dissolved in methanol and fixed to 10 mL to obtain a 1 mg/mL IS stock solution. For better peak shape of IS, the IS stock solution was diluted into 50 ng/mL of IS application working solution using acetonitrile. All solutions were stored at 4 degrees Celsius.

### 2.6. Plasma Sample Preparation

We used the protein precipitation method to prepare the samples. Briefly, after thawing the beagle dog plasma at room temperature, 50 *μ*L of plasma was withdrawn and 10 *μ*L of IS working solution (50 ng/mL) was added. The mixture was vortexed for 30 s, and then 200 *μ*L acetonitrile was added for precipitation. After vortex mixing for 1.0 min, the mixture was centrifuged at 15,000 rpm for 15 min, and, finally, 2 *μ*L of supernatant was taken into the UPLC-MS/MS system for detection.

### 2.7. Method Validation

The specificity, linearity, LLOQ, precision, accuracy, recovery, ME, and stability of the method were fully validated before the determination of duloxetine and 4-hydroxyduloxetine in beagle dogs plasma by this method. The UPLC-MS/MS method used in this study complies with the guidelines (Chinese Pharmacopoeia General Rules 9012) for validation of quantitative analysis methods for biological samples.

### 2.8. Plasma Sample Detection

The batch processing method was used, and the concentrations of duloxetine and 4-hydroxyduloxetine in the control group and experimental group were detected by the developed UPLC-MS/MS technique in this study. For samples whose concentration was higher than the upper limit of the standard curve, they needed to be diluted with blank plasma and then be detected again. The drug concentration was calculated based on the dilution factor.

### 2.9. Pharmacokinetics Study

The DAS (Drug and Statistics, version 2.0) was used to calculate the important pharmacokinetic parameters of duloxetine and 4-hydroxyduloxetine in the control group and experimental group through the statistical moment method; the actual measured values were used for peak concentration (*C*_max_) and peak time (*T*_max_). The main pharmacokinetic parameters of duloxetine and 4-hydroxyduloxetine were as follows: *C*_max_, *T*_max_, *t*1/2, CL, Vd, and AUC. Then the drug concentration-time curve was drawn.

### 2.10. Statistical Analysis

SPSS 16.0 software was used to compare the differences between the two groups; a *P* value less than 0.05 between groups indicated a statistical difference, and a *P* value less than 0.01 was considered a statistically significant difference.

## 3. Results

### 3.1. Selectivity

Three sets of samples were prepared: plasma from blank beagle dogs; plasma from beagle dogs plus with duloxetine, 4-hydroxyduloxetine, and IS; and plasma sample from beagle dogs after 3 h of oral administration of duloxetine hydrochloride enteric-coated tablets. Samples were processed and analyzed by UPLC-MS/MS, and the chromatograms were compared to determine whether endogenous substances were present in the plasma.

As shown in Figure 3 of the chromatogram, the endogenous substances in the plasma of beagle dogs did not affect the determination of duloxetine, 4-hydroxyduloxetine, and IS. The retention times of duloxetine, 4-hydroxyduloxetine, and IS were 1.29, 1.22, and 1.30 min, respectively. The smooth chromatographic baseline and good peak shape indicated that the UPLC-MS/MS method established in this experiment was specific and could meet the requirements of interaction detection.

### 3.2. Linearity

The plasma standards were prepared in triplicate at concentrations of 1, 5, 10, 50, 100, 250, 500, and 1000 ng/mL for duloxetine and concentrations of 0.1, 1, 2.5, 5, 10, 25, 50, and 100 ng/mL for 4-hydroxyduloxetine for three consecutive days. After processing, to calculate the linearity of each standard calibration curve, the relationship between the peak area ratio (Ai/as) and the analyte concentration was plotted.

A linear regression of the ratio of the drug peak area to the internal standard peak area (y) and the ratio of the drug concentration to the internal standard concentration (x) gave the regression equation for duloxetine: y = 4.73 × 10−3 x + 6.43 × 10−2 (r = 0.995 7), with LLOQ of 1 ng/mL. The regression equation for 4-hydroxyduloxetine is y = 6.9 × 10−3 x + 1 × 10−4 (r = 0.998 8), with LLOQ of 0.1 ng/mL. The LLOQ was defined as the lowest acceptable point in the standard curve.

### 3.3. Precision and Accuracy

The plasma standard solution was prepared at three concentration levels of duloxetine (2.5, 100, and 750 ng/ml) and three concentration levels of 4-hydroxyduloxetine (0.25, 10, and 75 ng/ml), with six samples prepared at each concentration (*n* = 6). The samples were analyzed on the same day to assess the intraday precision and accuracy and were analyzed for three consecutive days to calculate interday precision and accuracy. Precision was expressed as relative standard deviation (RSD, %) and was required to be less than 15%. Accuracy was expressed as a relative error (RE, %) and was required to be within ±15%

Table 3 shows the accuracy and precision results of duloxetine and 4-hydroxyduloxetine, from which it could be seen that the accuracy and precision values of duloxetine and 4-hydroxyduloxetine meet the requirements, with RSD ≤8.01% and RE between −1.33% and 2.85%.

### 3.4. Recovery and Matrix Effects (ME)

Duloxetine plasma standard samples were prepared at low, medium, and high concentrations (2.5, 100, and 750 ng/ml). Six samples were prepared in parallel for each concentration. Then the samples were treated according to the plasma sample preparation method, the samples were tested, and the peak area of duloxetine was recorded as A. Supernatants were extracted from six beagle plasma blanks, and three matrix controls with the same theoretical injection concentrations as the quality control were added to obtain the peak areas (B). The ratio of A to B was the extraction recovery. We evaluated the samples for matrix effect (ME). Ultra-pure water was used instead of blank plasma, and three reference solutions with the same concentration as the QC samples were added and analyzed to obtain the peak area (C). The MEs of duloxetine were calculated as B/C × 100%, respectively. In the same way, 4-hydroxyduloxetine plasma standard solutions were prepared at low, medium, and high concentrations (0.25, 10, and 75 ng/ml), and the recovery and ME of 4-hydroxyduloxetine were analyzed.

Table 4 demonstrates the recoveries and ME of duloxetine and 4-hydroxyduloxetine, from which it could be seen that the recoveries of duloxetine and 4-hydroxyduloxetine were more than 80%, and ME were near 100%. The ME did not affect the determination of duloxetine and 4-hydroxyduloxetine under the chromatographic and mass spectrometric conditions established in this study.

### 3.5. Stability

Quality control samples of three different concentrations of duloxetine (2.5, 100, and 750 ng/mL) and 4-hydroxyduloxetine (0.25, 10, and 75 ng/mL) were prepared with 6 parallel samples and treated according to the plasma treatment method described above and then subjected to four different environments (room temperature for 4 h, 4°C for 24 h, three cycles of freeze-thawing (-20 ∼ 25°C), and freezing at -80°C for 4 weeks).

The results of the stability of duloxetine and 4-hydroxyduloxetine under four conditions were shown in Table 5, from which it could be seen that the RE values of duloxetine and 4-hydroxyduloxetine ranged from −3.33% to 2.67% with RSD <10.93%. This indicates that duloxetine and 4-hydroxyduloxetine in the beagle dog samples were able to be stable under the four conditions mentioned above.

### 3.6. Pharmacokinetics of Duloxetine and 4-Hydroxyduloxetine

The plasma mean drug concentration-time profiles of duloxetine and 4-hydroxyduloxetine are shown in Figure 4. After DAS 2.0 analysis and processing, the pharmacokinetic parameters of duloxetine and 4-hydroxyduloxetine could be derived and are shown in Table 6.

### 3.7. Herb-Drug Interactions

After the coadministration of CHSGP with duloxetine hydrochloride, *C*_max_ and AUC_0⟶t_ of duloxetine decreased by 49.33% and 13.08%, respectively, *T*_max_ was significantly prolonged, and *t*_1/2_ was shortened to 10.17 h. The results indicated that CHSGP delayed the absorption of duloxetine, decreased plasma exposure, and induced its metabolism. Meanwhile, after the coadministration of CHSGP with duloxetine hydrochloride, *C*_max_ and AUC_0⟶t_ of 4-hydroxyduloxetine decreased by 71.47% and 48.78%, respectively, *T*_max_ was significantly prolonged, the CL increased significantly, and *t*_1/2_ was shortened to 7.97 h. The results indicated that CHSGP decreased the plasma exposure of 4-hydroxyduloxetine and induced the metabolism of 4-hydroxyduloxetine.

## 4. Discussion

### 4.1. Method Validation and Improvement

The main methods used to detect duloxetine hydrochloride were HPLC [13] and LC-MS [14–16]. UPLC-MS/MS technology was a common method for drug-drug interactions (DDIs) and herb-drug interactions (HDIs) [17–19](Ruan et al.; Xia et al., 2021; Zhu et al., 2019). So, in this study, we optimized the methodology according to the concept and principles of Green Analytical Chemistry (GAC) [20] and established a UPLC-MS/MS for the simultaneous determination of duloxetine as well as its metabolite 4-hydroxyduloxetine in beagle dog plasma. From the methodological data, it was evident that the method was highly sensitive and detected concentrations as low as 1 ng/mL (duloxetine) and 0.1 ng/mL (4-hydroxyduloxetine), respectively. The analysis time was only 2 min, which was suitable for the analysis of large volume samples.

For the plasma clean-up, protein precipitation with acetonitrile was used, which is simple to operate compared with solid phase extraction and liquid-liquid extraction, resulting in a high recovery with no matrix effect. As for the choice of IS, we compared diazepam, fluoxetine, and paroxetine under the existing laboratory conditions, and the results showed that when the IS was fluoxetine, it had a good separation from duloxetine and 4-hydroxyduloxetine with good peak shape, similar peak times, and similar recoveries and was not interfered by endogenous substances in the plasma of beagle dogs.

### 4.2. Drug-Drug Interaction

Drug-drug interaction was broadly defined as the physical and chemical changes that occurred between two or more drugs in vitro and the changes in pharmacological effects that result from these changes in vivo

In a narrower sense, it referred to the changes in pharmacokinetics and pharmacodynamics between drugs in vivo, which included changes in the strength of the effect (enhancement or weakening), as well as changes like the action (ineffectiveness or toxicity) that may affect the efficacy and safety of the drug application.

Rational drug interactions could enhance efficacy or reduce adverse drug reactions and conversely could lead to reducing efficacy or increasing toxicity, as well as some abnormal reactions that could interfere with treatment and aggravate the condition.

Our previous research results showed that Danzhi Xiaoyao pills can accelerate the metabolism of venlafaxine in beagle dogs, reduce the plasma exposure of venlafaxine, and increase the content of O-desmethylvenlafaxine (ODV) and N-desmethylvenlafaxine (NDV) [19]. Sijunzi Pills could inhibit the metabolism of omeprazole and increase the concentration of omeprazole in beagle dogs [18].

In this experiment, CHSG was given to beagle dogs for 15 consecutive days, which was sufficient for CHSG to reach steady-state blood concentrations and to affect liver drug enzymes in vivo. The significant changes in the concentrations of both duloxetine and its metabolites occurred after the coadministration with CHSG, indicating that CHSG could affect the metabolism of duloxetine. Both duloxetine and 4-hydroxyduloxetine were metabolized through CYP1A2 and CYP2D6, and the increase in enzyme activity caused a decrease in the amount of duloxetine and a decrease in metabolite content. Therefore, CHSG was able to induce the metabolism of duloxetine and its metabolites in beagle dogs.

It had been reported that peony can induce CYP1A2 enzyme activity and increase CYP1A2 enzyme gene mRNA expression, and glycyrrhetinic acid and glycyrrhizin in licorice had an inductive effect on CYP1A2 gene expression and the mixed components of licorice could induce the expression of CYP2D6. So, we speculate that the induction of metabolism of duloxetine and its metabolites by CHSG in this study may be due to the increase of CYP1A2 or CYP2D6 activity by some components in CHSG, but whether the changes are caused by modulation of enzyme activity needs to be verified by in vitro liver microsomal experiments.

## 5. Conclusions

The successfully developed UPLC-MS/MS method for the simultaneous determination of duloxetine and its metabolite 4-hydroxyduloxetine was fast, sensitive, and stable, and the methodological data met the pharmacokinetic requirements. CHSG could slow down the absorption of duloxetine and at the same time reduce the plasma exposure of duloxetine and its metabolites, that is, induce the metabolism of duloxetine. Based on the possibility of this result, it was recommended that the dose should be adjusted when CHSG is combined with duloxetine in clinical practice.

## Figures and Tables

**Figure 1:** Information on components in CHSG. (a) Figures of herbs in CHSG. (b) Ratio of each herb in CHSG.

**Figure 2:** The chemical structure of duloxetine (a) and 4-hydroxyduloxetine (b).

**Figure 3:** Chromatograms of duloxetine and its metabolite 4-hydroxyduloxetine. (a) Blank beagle dog plasma; (b) a blank beagle dog plasma spiked with duloxetine, 4-hydroxyduloxetine, and IS; (c) a plasma sample from a beagle dog.

**Figure 4:** The average plasma drug concentration-time curve of duloxetine (a) and 4-hydroxyduloxetine (b) in beagle dogs (*n* = 6).

**Table 1:** The Chinese, herbal, and botanical names of the corresponding herb in CHSG.

Chinese name	Herb name	Botanical name	Ratio (%)
Chai-hu	Radix bupleuri	*Bupleurum* Chinese DC.	19.05
Chen-pi	Pericarpium citri reticulatae	*Citrus reticulata* Blanco	19.05
Chuanxiong	Rhizoma chuanxiong	*Ligusticum chuanxiong* Hort.	14.29
Xiang-fu	Rhizoma cyperi	*Cyperus rotundus* L.	14.29
Zhi-qiao	Fructus aurantii	*Citrus aurantium* L.	14.29
Shao-yao	Chinese herbaceous peony	*Paeonia lactiflora* Pall.	14.29
Zhi-gan-cao	Roasted licorice	*Glycyrrhiza uralensis* Fisch.	4.76

**Table 2:** UPLC Gradient elution procedures.

Time (min)	Flow rate (mL/min)	0.1% formic (%)	Acetonitrile (%)
0	0.4	90	10
0.5	0.4	90	10
1.0	0.4	10	90
1.4	0.4	10	90
1.5	0.4	90	10
2.0	0.4	90	10

**Table 3:** Precision and accuracy of duloxetine and 4-hydroxyduloxetine in beagle dog plasma (*n* = 6, Mean ± SD).

Analytes	Added (ng/mL)	Intraday				Interday	
		Mean ± SD	RSD (%)	RE (%)	Mean ± SD	RSD (%)	RE (%)
Duloxetine	2.5	2.53 ± 0.20	8.01	1.18	2.48 ± 0.19	7.73	-0.61
	100	99.43 ± 7.58	7.62	-0.58	101.03 ± 6.30	6.23	1.03
	750	742.22 ± 25.38	3.42	−1.04	753.09 ± 31.82	4.22	0.41
4-Hydroxyduloxetine	0.25	0.247 ± 0.02	7.97	−1.33	0.256 ± 0.02	7.85	2.22
	10	10.29 ± 0.70	6.76	2.85	9.96 ± 0.60	6.04	-0.37
	75	75.13 ± 2.44	3.25	0.17	75.58 ± 2.80	3.71	0.78

**Table 4:** Recoveries and ME of duloxetine and 4-hydroxyduloxetine in beagle dog plasma.

Analytes	Added (ng/mL)	Recovery (%)	RSD (%)	ME (%)	RSD (%)
Duloxetine	2.5	81.53 ± 2.56	3.14	98.35 ± 4.56	4.64
	100	83.73 ± 4.09	4.89	101.64 ± 4.95	4.87
	750	84.05 ± 3.06	3.65	102.57 ± 4.08	3.98
4-Hydroxyduloxetine	0.25	79.97 ± 3.66	4.57	102.62 ± 4.02	3.91
	10	80.73 ± 4.46	5.53	98.88 ± 4.46	4.51
	75	82.24 ± 3.05	3.71	101.44 ± 4.30	4.24

**Table 5:** Stability results of duloxetine and 4-hydroxyduloxetine in beagle dog plasma in different conditions.

Analytes	Added (ng/mL)	Room temperature, 4 h		Autosampler 4°C, 6 h		Three freeze-thaw		−20 °C, 4 weeks	
		RSD (%)	RE (%)	RSD (%)	RE (%)	RSD(%)	RE(%)	RSD(%)	RE(%)
Duloxetine	2.5	8.16	−3.07	9.59	2.47	6.39	−1.73	8.65	1.80
	100	4.61	1.05	6.91	−0.36	4.54	1.34	3.79	−1.79
	750	3.88	1.16	4.76	0.81	3.93	-0.73	1.72	0.61
4-Hydroxyduloxetine	0.25	8.84	−3.33	10.93	2.67	6.71	−2.00	6.45	1.33
	10	4.33	1.37	6.69	−0.15	4.61	1.18	3.79	−1.73
	75	3.31	1.08	4.74	0.84	3.85	−0.68	2.40	0.27

**Table 6:** The main pharmacokinetic parameters of duloxetine and 4-hydroxyduloxetine in the control and experimental group (*n* = 6, mean ± SD).

Parameters	Duloxetine		4-Hydroxyduloxetine	
	Control group	Experimental group	Control group	Experimental group
*t*_1/2_ (h)	13.58 ± 4.26	10.17 ± 3.01^*∗*^	11.23 ± 1.79	7.97 ± 2.05^*∗*^
*T*_max_ (h)	1.17 ± 0.26	3.50 ± 1.38^*∗∗*^	1.67 ± 0.26	4.33 ± 1.51^*∗∗*^
MRT_(0-t)_ (h)	5.37 ± 1.10	7.37 ± 2.17^*∗*^	7.73 ± 0.81	9.60 ± 2.40^*∗*^
MRT_(0-∞)_ (h)	7.03 ± 1.63	8.39 ± 1.86	9.02 ± 1.26	10.32 ± 2.49
*C*_max_ (ng/mL)	469.14 ± 185.61	237.70 ± 95.13^*∗∗*^	47.70 ± 19.83	13.48 ± 7.07^*∗∗*^
CLz/F (L/h/kg)	1.75 ± 0.69	2.02 ± 0.68	13.41 ± 8.34	25.39 ± 15.25^*∗∗*^
AUC_(0-t)_ (ng·h/mL)	1262.10 ± 467.36	1096.96 ± 463.92	178.37 ± 70.00	92.57 ± 31.31^*∗∗*^
AUC_(0-∞)_ (ng·h/mL)	1291.33 ± 466.82	1113.04 ± 461.70	183.29 ± 71.06	93.88 ± 31.49^*∗∗*^

*Note.* Compared with the control group, ^*∗*^*P* < 0.05 and ^*∗∗*^*P* < 0.01.

## Data Availability

The original contributions presented in the study are included within the article and further data can be obtained from the corresponding author upon request.
